This article has been retracted.

# Multidimensional CNN-Based Deep Segmentation Method for Tumor Identification

**DOI:** 10.1155/2022/5061112

**Published:** 2022-08-21

**Authors:** R. John Martin, Uttam Sharma, Kiranjeet Kaur, Noor Mohammed Kadhim, Madonna Lamin, Collins Sam Ayipeh

**Affiliations:** ^1^Faculty of Computer Science and Information Technology, Jazan University, Saudi Arabia; ^2^Department of Computer Science and Engineering, Gautam Buddha University, Greater Noida, India; ^3^Department of CSE, University Centre for Research & Development, Chandigarh University, Mohali, Punjab 140413, India; ^4^Department of Medical Instruments Engineering Techniques, Al-Farahidi University, Baghdad 10021, Iraq; ^5^Computer Science and Engineering, ITM SLS Baroda University, Vadodara, 391510 Gujarat, India; ^6^Kwame Nkrumah University of Science and Technology, Kumasi, Ghana

## Abstract

Weighted MR images of 421 patients with nasopharyngeal cancer were obtained at the head and neck level, and the tumors in the images were assessed by two expert doctors. 346 patients' multimodal pictures and labels served as training sets, whereas the remaining 75 patients' multimodal images and labels served as independent test sets. Convolutional neural network (CNN) for modal multidimensional information fusion and multimodal multidimensional information fusion (MMMDF) was used. The three models' performance is compared, and the findings reveal that the multimodal multidimensional fusion model performs best, while the two-modal multidimensional information fusion model performs second. The single-modal multidimensional information fusion model has the poorest performance. In MR images of nasopharyngeal cancer, a convolutional network can precisely and efficiently segment tumors.

## 1. Introduction

Nasopharyngeal carcinoma (NPC) is the most common malignant tumor in the human nasopharynx. According to the World Health Organization report, about 80% of NPC patients worldwide are concentrated in China, and most of the remaining patients are found in Southeast Asia and the Middle East and North Africa [1, 2]. According to statistics, the incidence of NPC in Guangzhou is 17.8 per 100,000 people, the incidence rate is rising, and the incidence is younger [3]. However, most patients have missed the most. Therefore, the early diagnosis of NPC is essential to seize the best time for treatment. At present, the treatment of NPC is mainly radiotherapy, and the accurate localization of NPC lesions is a crucial basis for the formulation of radiotherapy plans and implementation of radiotherapy. In radiation therapy, high-energy X-rays are utilized to destroy cancer cells. A schedule for radiation therapy normally consists of a certain number of sessions spaced out over a defined period of time. The most common form of external beam radiation therapy used to treat NPC sends radiation from a machine outside the body directly at the tumor. With the reduced risk to healthy cells and fewer side effects, intensity-modulated radiation therapy, a kind of external beam radiation therapy, makes it possible to administer larger radiation therapy doses. The ASCO suggests intensity-modulated radiation therapy for all patients with stage II to stage IVA NPC.

NPC segmentation is a difficult procedure since the morphological structure of the nasopharyngeal region is convoluted, the severity of the tumor is equivalent to that of neighboring tissues, and the morphology of the tumor varies greatly across individuals. Traditional manual tumor contour segmentation, a crucial step in radiotherapy, has become labor- and time-intensive due to the enormous amount of data produced by several patients. As a result, there is an increasing need for automated segmentation algorithms that are trustworthy in order to lighten the workload of radiologists. MR images are often used in diagnosing and localization of NPC due to their high resolution and strong safety. Before making a treatment plan, clinicians usually need to examine each MR image. Whether there is a lesion in the image and manually outline the tumor boundary, due to the complex and changeable shape, size, and location of the tumor between different NPC patients, this process has disadvantages such as heavy workload, high requirements for doctors' experience, and significant subjective influence. Therefore, researchers have sought to delineate the NPC lesion area automatically. The cancer care team will suggest a treatment plan based on the kind, severity, and extent of the nasopharynx cancer as well as its stage and rate of spread. The conventional therapy for these early-stage cancers is radiation therapy focused on the tumor. Although radiotherapy is frequently used to treat the neck's surrounding lymph nodes, cancer has not yet spread to the lymph nodes at this time. Stages II, III, IVA, and IVB patients with varying stages of NPC typically get chemotherapy to the nasopharynx and neck lymph nodes. In addition to the targeted drug cetuximab, chemotherapy is frequently used to treat patients with stage IVC (Erbitux). Another alternative is immunotherapy.

Traditional image segmentation approaches, such as the threshold method, area growth method, and statistical theory [4, 5], as well as machine learning methods, such as support vector machines and artificial neural networks [6, 7], are used to segment NPC tumors. The threshold is a well-liked method of segmenting images. It aids in separating the backdrop from the foreground. By selecting the proper threshold value T, the grey level photograph may be converted into a binary image. The binary image should fully expose the elements of interest's orientation and structure (foreground). Getting a binary image from the outset has the advantage of reducing complexity and simplifying the identification and verification procedures.

Deep learning is a crucial diagnostic technology that produces accurate findings by using an organized network with homogeneous portions. Utilizing statistical model automatic segmentation approaches in several essential scenarios, its excellent quality has been shown. Performance measurements demonstrate that deep learning algorithms are significantly more successful at segmenting pictures than a statistical method. For a number of diverse medical image segmentation tasks, the deep learning approach is applied with the highest level of accuracy. The process of segmenting pictures will need the development and comparison of a number of deep learning algorithms in the future.

The SVM model can function by choosing an appropriate margin or hyperplane when there are values in the characteristics of two groups that tend to group around distinct values, such as predicting values associated with a tumor grade or categorizing various tissues with varied attenuation and textures exhibited. Support vector machines have been used successfully to solve problems with image segmentation and classification. Early image segmentation algorithms were built on digital image processing and optimization approaches.

With the help of methods like region growth and the snake's algorithm, which included creating beginning regions, these early algorithms compared pixel values to get an understanding of the segment map. These methods took a localized view of an image's characteristics by focusing on local gradients and pixel differences. Edge detection, Otsu's algorithm, and clustering algorithms were developed somewhat later among the common image processing techniques. These algorithms viewed the input image from a broad perspective. Such ideas almost always need the inclusion of features. Manual intervention procedures like extraction and dimensionality reduction have drawbacks like model robustness and noise sensitivity. Less time and storage space are required with dimensional reduction. It helps eliminate multicollinearity, improving comprehension of the machine learning model's parameters. It removes those features from the data since including irrelevant features in the data might decrease model accuracy and cause your model to train using irrelevant traits.

As a result, adopting such approaches to create quick automated segmentation of NPCs is difficult. Convolutional neural networks (CNN) and other deep learning (DL) approaches have been extensively employed in medicine. Segmenting an item that may be moved in the image is extremely difficult since the CNN model is not scale- and rotation-invariant. The speed of evaluation is one of the main issues with employing a CNN model in the medical field, as many pharmacological treatments require quick replies to reduce the need for extra investigation and treatment. They can extract characteristics in pictures directly and automatically, from low-level to high-level, abstract to concrete. Image classification, segmentation, and registration are all techniques used in image processing. Literature [8] employed an encoder-decoder fully convolutional neural network to segment CT images of NPC patients and compared it to the VGG network [9] in NPC segmentation. The findings suggest that the network can significantly enhance NPC segmentation.

Literature [10] employed a fully convolutional neural network with an encoder-decoder to segment the MR images of 27 NPC patients and used leave-one-out cross-validation to accomplish NPC segmentation. Literature [11] also employed a convolutional neural network to separate the lesion region of 30 NPC patients' T1W modality MR data. To enhance the segmentation findings, they applied a 3D graph cut technique. The value of the Dice is 0.851. All of the models utilized in the preceding experiments are 2D models. As a result, the association of visual characteristics in 3D space is not taken into account. 2D CNN typically achieves higher Dice scores than its 3D version for three reasons: first, if we opt to work with volumes above slices for a particular data set of 3D pictures, the sample size is less, which may cause convergence issues during network training. Second, we can increase the output of a 2D design greater than its 3D version for a given set of computer resources. When deep learning architectures are designed for 2D pictures, 3D data offers various challenges, such as less effective volumetric input pipelines. Third, 3D image processing requires extra code since image augmentation libraries were created for 2D pictures. Additionally, working with volumes calls for greater processing power, particularly RAM and VRAM. The network topology is basic, the experimental data is limited, and segmentation is limited to pictures from a single modality. However, since the local knowledge of NPC tumors represented by single-modality imaging data is restricted, the model's resilience must be increased.

Even though the 2D network has fewer parameters and can fit models quickly, it does not properly utilize the topological information between layers. As a consequence, the segmentation results are prone to inaccuracy and irregular borders [12]. The 3D network may compensate for this shortcoming, but it comes with the drawbacks of a large number of parameters and sluggish or even difficult model fitting. As a result, this work integrates 2D and 3D information using the H-DenseUNet model suggested by literature [13]. To assist doctors in the diagnosis and treatment planning of hepatocellular carcinoma, an accurate and computerized liver and tumor segmentation strategy is highly sought in clinical practice. However, 2D convolutions are constrained in their capacity to effectively exploit location data along the third dimension, whereas 3D convolutions suffer from a severe computational expense and GPU memory usage. To address these issues, a brand-new hybrid densely linked UNet (H-DenseUNet) is proposed. It is made up of a 2D DenseUNet for efficiently extracting intraslice characteristics and a 3D counterpart for hierarchically aggregating volumetric contexts, similar to how the autocontext algorithm segments tumors and the liver. Specifically, the 2D network's quick segmentation findings are utilized to drive the 3D model's learning and implementation of segmentation [14]. A new deep segmentation method of multimodal and multidimensional information fusion is proposed using MR images of three modalities, T1W, T2W, and T1C, to establish a multimodal 2D-ResUNet 3D-ResUNet multidimensional feature fusion model to achieve automatic and accurate segmentation of NPC lesions.

## 2. Research Method

### 2.1. Network Structure

Figure 1 depicts the deep convolutional neural network structure, which primarily consists of a multimodal 2D-ResUNet system, 3D-ResUNet structure, and 2D+3D fusion layer. A 3D picture I R13844384b3 is used as the model's input. The batch size, image height (*h*), image width (*w*), image depth (*b*), and numerous picture channels (*c*) of the input network are all represented by the size 1384384b3. The picture modalities T1W, T2W, and T1C are represented by the number of image channels *c* = 3.

First, three modalities of 2D pictures are produced if the function defines the process of transforming 3D images into 2D and explains the inverse operation of the transformation; second, the 2D network is defined as after multimodal 2D-ResUNet, the feature map and probability map of the 2D image is as follows:

(1) $$\begin{array}{c} F_{2d}=f_{2d}\left(I_{2d-T1W},I_{2d-T2W},I_{2d-T1C};\theta_{2d}\right),\;F_{2d}\in R^{b*384*384*16},\\ y_{2d}=f_{2dcls}\left(F_{2d};\theta_{2dcls}\right),y_{2d}\in R^{b*384*384*2}. \end{array}$$

The parameters of the convolutional network and the classification network, respectively, are *θ*_2*d*_ and *θ*_2*dcls*_ in the formula. *F*_2*d*_ and *y*_2*d*_ must perform the following inverse transformations to get the relevant 3D feature map to merge the findings of the 2D network with the 3D web:

(2) $$\begin{array}{c} {\hat{F}}_{2d}=T^{-1}\left(F_{2d}\right),\;{\hat{F}}_{2d}\in R^{1*384*384*b*16},\\ {\hat{y}}_{2d}=T^{-1}\left(y_{2d}\right),\;{\hat{y}}_{2d}\in R^{1*384*384*b*2}. \end{array}$$

Merge ${\hat{y}}_{2d}$ with *I* and input them into 3D-ResUNet to get the feature map of the 3D network:

(3) $$\begin{array}{c} F_{3d}=f_{3d}\left(I,{\hat{y}}_{2d};\theta_{3d}\right),F_{3d}\in R^{1*384*384*b*16}. \end{array}$$

In the formula, *θ*_3*d*_ is the parameter of the 3D network. After summing ${\hat{F}}_{2d},F_{3d}$ to get *Z*, input the 2D+3D fusion layer *f*_*HF*_, perform convolution calculation to get *H*, and then go through the classification layer *f*_*HFcls*_ to get the 3D segmentation result *y*_*H*_.

(4) $$\begin{array}{c} Z={\hat{F}}_{2d}+F_{3d},\\ H=f_{HF}\left(Z;\theta_{HF}\right),\\ y_{H}=f_{HFcls}\left(H;\theta_{HCFcls}\right). \end{array}$$

The parameters of the convolutional layer *f*_*HF*_ of the fusion layer and the classification layer *f*_*HFcls*_, respectively, are represented by the formula: HF and HFcls. We are aware that the network aims to recognize the fundamental patterns in each Conv Layer. For instance, the network attempts to learn patterns and edges in the first layer. It tries to comprehend the form, color, and other things in the second layer. The picture is attempted to be classified by a final layer known as the feature layer or fully connected layer. The first fully connected layer, which is a convolutional layer and presents the last challenge in the CNN layer, is unknown in terms of its dimensions. The size of each convolution layer must first be determined, starting with the size of the input picture.

Table 1 shows the network architecture and associated parameters for 2D-ResUNet and 3D-ResUNet. The model is built using the ResUNet with residual structure because the residual design may effectively tackle issues like gradient disappearance [15]. It is employed in activities involving computer vision. It has been shown that the performance of the network is superior to that of a network with convolutional layers stacked on top of each other [16]. The network combines the benefits of the 2D network's quick fitting speed with the 3D grid's adequate use of spatial information. It employs the 2D web segmentation findings to drive the fitting of the 3D model, allowing for more efficient model training and testing.

### 2.2. Multimodal 2D Convolution

The multimodal 2D-ResUNet structure is shown in Figure 2, which mainly includes an encoder of three modal images, a multimodal convolution structure, a decoder, and a skip connection structure between the encoder and the decoder. The decoder consists of a convolution block with residual structure and a deconvolution layer. Each pooling layer pools the three modal images in the encoder [17]. And then, perform the convolution operation on the three types of feature maps after pooling to realize the fusion of multimodal 2D features. The specific implementation process is as follows: the three modal images undergo the same level of convolution and pooled feature maps. With the same size, by merging the three feature maps in the direction of the image depth, a 3D feature map with a depth of 3 can be generated [18]. Then, a convolution kernel of size (1, 1, 3) is used to create a (1, 1, 3). Convolve the feature map for the step size so that the depth of the feature map is converted to 1, and the profound fusion of the three modal features is realized. Finally, the same filter level feature maps are added to reduce the loss of information in the deconvolution process.

### 2.3. Multimodal 3D-ResUNet

*y*_2*d*_ T^−1^ by ${\hat{y}}_{2d}$ is shown in Figure 1. The input of the multimodal 3D-ResUNet is the image obtained after the transformation of the segmentation probability map of the multimodal 2D-ResUNet and the original information of the model, so the input size is 1 × 384 × 384 × b × 5, where “5” means that the network input is 5 channels, which are 3 modal images and the segmentation probability map of tumor and background obtained by the multimodal 2D-ResUNet network. 3D segmentation can be achieved by inputting the 3D-ResUNet network with skip connections and residual structure [19]. Therefore, the network uses 3 modal images as the three channels of the input image and the multimodal 2D-ResUNet segmentation probability map as input two tracks of the image; thus, using the 2D network fast segmentation results to guide 3D model segmentation.

The suggested MultiRes block is used to replace the series of two convolutional layers in the MultiResUNet model. The 18-layer ResNet CNN is chosen above the other CNNs because it has a greater accuracy and requires fewer compute processes.  Figure 2 depicts the algorithm's structure. A 7 × 7 kernel filter with a stride of 2 first filters the input picture to 64 channels. 3 × 3 kernel filters convolute the remaining blocks. The skip connection arrow connects the two blocks to avoid gradients vanishing, which is the ResNet algorithm's fundamental competency.

### 2.4. Loss Function Calculation

The Sorensen-Dice coefficient is a statistic created in the 1940s to assess the similarity between the two samples, which is where Dice loss gets its name. Milletari et al. presented it to the computer vision community in 2016 for 3D medical picture segmentation. The ground truth border pixels and anticipated boundary pixels in boundary detection tasks may be seen as two sets. The two sets are programmed to gradually overlap by using Dice loss. Due to the importance of high accuracy, Dice loss takes into account the loss of data both locally and internationally. In the MR images of nasopharyngeal carcinoma patients in this study, the proportion of the tumor area relative to the entire image is tiny; that is, the size of the tumor area is much smaller than the area of the nontumor site, so the Dice loss [20] is used as the primary loss function, defined as follows:

(5) $$\begin{array}{c} \text{Dice}=\frac{2\left|P\cap G\right|}{\left|P\right|+\left|G\right|}. \end{array}$$

In the formula, *P* is the output result of the model, and *G* is the actual label, that is, the manually drawn tumor contour.

Dice loss is defined as

(6) $$\begin{array}{c} L=1-\text{Dice}. \end{array}$$

The total loss of the model consists of two parts: the loss *L*_2D_ of 2D-ResUNet and the loss *L*_*F*_ of the 2D+3D fusion layer. Therefore, the complete loss of the model is the weighted sum of these two losses:

(7) $$\begin{array}{c} L_{\text{Total}}=\alpha L_{2\text{D}}+L_{F}. \end{array}$$

In the formula, *α* is the weight of 2D-ResUNet loss, which is set to 0.5 in this study, indicating that the model pays more attention to the loss of the final output.

## 3. Data Set

421 NPC patients were collected with T1W, T2W, and T1C MR images of three brain structures, and 1.5T GE Medical Systems was used for horizontal scanning. The MR image has TE = 8.69 ms, DFOV = 198 mm, slice thickness 6 mm and total of 31 slices. T1C image parameters are TR = 753 ms, TE = 8.69 ms, DFOV = 198 mm, and slice thickness 6 mm; there are 31 layers in full; the parameters of the T2W image are TR = 2900 ms, TE = 83.56 ms, and DFOV = 189 mm, the layer thickness is 5 mm, there are 32 layers in total, and the resolution of all 3D image horizontal slices is 512 × 512. An experienced clinician manually delineated the tumor region of the T2W modality images to determine the segmentation labels. The images of 346 patients were randomly selected from all 421 subjects as the training set. The images of the remaining 75 patients were used as the independent test set; the information on the training set and test set is shown in Table 2.

## 4. Experimental Result Analysis

### 4.1. Evaluation Indicators

The Dice coefficient [5], Hausdorff distance (HD) [5], and percentage of area difference (PAD) [6] are used as the evaluation indicators of the model effect. HD and PAD are defined as follows:

(8) $$\begin{array}{c} \text{HD}\left(P,G\right)=\underset{a\in P}{\max}\left\{\underset{b\in G}{\max}\left[d\left(a,b\right)\right]\right\}, \end{array}$$

where *d*(*a*, *b*) is the Euclidean distance.

(9) $$\begin{array}{c} PAD=\frac{\left|P-G\right|}{G}. \end{array}$$

The smaller the values of HD and PAD, the closer the model segmentation results are to the manual delineation results, and the better the model performance.

### 4.2. Training and Testing

Firstly, the single-modal multidimensional fusion models of T1W, T2W, and T1C three modal data were constructed by using single-modal 2D-ResUNet and 3D-ResUN et and 2D+3D fusion layers, respectively, which are T1W-MDF, T2W-MDF, T1C-MDF; then, combine T1W, T2W, and T1C in pairs, namely, T1W+T2W, T1W+T1C, and T2W+T1C, a total of three dual-modal images as two channels of the 3D image, respectively, to recombine the 3D image. Then, the 2 modal images are used as the input of each encoder of the mmultimodal2D-ResUNet, and the 2D-ResUNet output probability map and the 2 modal 3D input images are merged and then input into 3D-ResUNet and then passed through 2D+3D. The fusion layer constructs two-modal multidimensional information fusion segmentation models, which are T1W+T2W-MDF, T1W+T1C-MDF, and T2W+T1C-MDF; finally, the three modal images of T1W, T2W, and T1C are used as the 3D images, respectively. Three-channel, after the 3D image is reorganized, each modal image is used as the input of each encoder of the mmultimodal2D-ResUNet, and the output probability map of the mmultimodal2D-ResUNet is combined with the mmultimodal3D input image. After merging, they are input into 3D-ResUNet, and then, a multimodality multidimensional fusion (MMMDF) segmentation model is constructed through a 2D+3D fusion layer.

The TensorFlow [21] software library is used to build the model. The initial learning rate in the training phase is 0.001, and the attenuation is multiplied by 0.9 every 4 rounds. The Adam optimizer is used for optimization. The graphics card is NIVIDIA Titan XP GPU, a single-modal multidimensional fusion model, dual-mode. The training time of the multimodal fusion model and the multimodal fusion model was 23 h 37 min, 30 h 24 min, and 34 h 47 min, respectively. The testing time of each patient in the three types of models in the testing phase was about 13, 18, and 18 minutes, respectively—22 s.

Using the same training set and test set, the algorithms in the literature [8, 10, 16] are trained and tested, and the results are compared with the MMMDF method proposed in this paper, as shown in Table 3. For the different models in this paper, the resulting boxplot is shown in Figure 3.

It can be seen from Table 2 and Figure 3 that the segmentation performance of the MMMDF model is better than that of the model with any single modality of T1W, T2W, and T1C as input and better than any two-modal multidimensional fusion segmentation model. The MMMDF segmentation results are compared with 3. A statistical test was carried out on the segmentation results of the two-modal multidimensional fusion. The results showed that the *P* values of the Dice coefficient, the area difference ratio, and the Hausdorff distance were all less than 0.05, indicating that the segmentation performance of the MMMDF model was better than that of any two-modal multidimensional fusion model. Calculating the average Hausdorff distance between the two-point sets is a typical practice evaluation metric. In medical image segmentation, it is utilized to compare actual photos to the segmentations that allow for their ranking. The Dice coefficient and the IoU have many similarities. They are positively correlated, so if one asserts that model A is better at segmenting pictures than model B, the other will do the same. Similar to the IoU, they also have a range from 0 to 1, with 1 being the maximum similarity between predicted and truth. The Dice coefficient should ideally not be higher than 1. A Dice coefficient typically ranges from 0 to 1. If you are obtaining a coefficient greater than 1, perhaps, you should check your implementation. The performance is better and has statistical differences. Using multimodality as the input of 2D-ResUNet, in the process of network convolution, the information of different modalities is fused: in addition, multimodal images are used as the input of 3D-ResUNet, and the communication between other modalities is connected again, so the effect of the fusion model is better than the effect of single-modal intake. In addition, the use of multidimensional models in series combines the fast-fitting speed of 2D models and the characteristics of 3D models. After learning the good advantages, a better segmentation effect is obtained on the test set.

It can be seen from Table 2 that compared with the methods mentioned in other literature, the MMMDF segmentation model proposed in this paper has a significant improvement in the performance of NPC segmentation. This is because the studies in this literature only use a simple 2D encoder-decoder network or fine-tune the network structure based on this while only taking a single modality image.

Figure 4 shows the partial segmentation results obtained by the T1W-MDF, T2W-MDF, T1C MDF, and MMMDF models. Morphology, volume, and tumors in different regions showed excellent segmentation results. In Figures 4 and 5, each row represents another patient, and the first column represents the input image; the 2~8 columns represent T1W-MDF, T2W, the methods of MDF, T1C-MDF, Methods1 [20], Methods2 [15], and Methods3 [22], and the results of MMMDF. The first column of Figure 4 is the final image, and the second to eighth columns are the enlarged images of the first column of the window area. Two lines represent the manually delineated tumor region (gold standard) and the model segmentation result. The performance comparison of different NPC segmentation models is shown in Table 3.

## 5. Conclusion

This work used three modal MR scans of T1W, T2W, and T1C of the head and neck of NPC patients to obtain precise segmentation of lesions in NPC patients. It developed a novel deep learning segmentation model based on multimodal and multidimensional information fusion. In the experiment, the findings reveal that the multimodal multidimensional information fusion model can more correctly detect lesions and enhance the segmentation effect when compared to the single-modal multidimensional fusion model and other existing approaches for NPC lesion segmentation. The approach suggested in this study may efficiently and accurately localize NPC tumors, offer an objective foundation for NPC diagnosis and therapy, and increase the efficiency and level of diagnosis and treatment. This research contains four major flaws: (1) a total of 421 patients' MR pictures were obtained in three modalities, with a modest number of patient samples. (2) The resolution is poor, the slice thickness is 5 mm, and the spatial structure information is discontinuous or partly absent; therefore, increasing the sample size will assist in enhancing the segmentation model's generalization capacity. On the one hand, it makes identifying the tumor location in the training sample more challenging. On the other hand, it prevents the 3D segmentation model from making efficient use of the image's layer topological information. (3) The model's segmentation performance is poor in certain tumor locations with a small area, and it is required to concentrate on how to improve the segmentation results by using tumor area information from neighboring layers. (4) Different modal pictures have different positions. Space is guaranteed. The model's dependability and flexibility will benefit from the regular position.

## Figures and Tables

**Figure 1:** Convolution neural network structure with multimodal and multidimensional fusion.

**Figure 2:** Multimodal 2D-ResUNet structures.

**Figure 3:** Comparison of performance box plots of seven NPC segmentation models.

**Figure 4:** Comparison of the 2D segmentation results.

**Figure 5:** Comparison of the 3D segmentation results.

**Table 1:** 2D-ResUNet and 3D-ResUNet network structures.

Network layer	2D-ResUNet		3D-ResUNet	
	Feature map size	Network layer size	Feature map size	Network layer size
Input	384 × 384	—	384 × 384 × 8	—
Residual structure 1	384 × 384	[3 × 3, 16] × 5	384 × 384 × 8	[3 × 3 × 3, 16] × 5
Max pooling layer 1	192 × 192	2 × 2 max pooling	192 × 192 × 4	2 × 2 × 2 max pooling
Residual structure 2	192 × 192	[3 × 3, 32] × 5	192 × 192 × 4	[3 × 3 × 3, 32] × 5
Max pooling layer 2	96 × 96	2 × 2 max pooling	96 × 96 × 4	2 × 2 × 1 max pooling
Residual structure 3	96 × 96	[3 × 3, 64] × 5	96 × 96 × 4	[3 × 3 × 3, 64] × 5
Max pooling layer 3	48 × 48	2 × 2 max pooling	48 × 48 × 2	2 × 2 × 2 max pooling
Residual structure 4	48 × 48	[3 × 3, 128] × 5	48 × 48 × 2	[3 × 3 × 1, 128] × 5
Max pooling layer 4	24 × 24	2 × 2 max pooling	24 × 24 × 2	2 × 2 × 1 max pooling
Residual structure 5	24 × 24	[3 × 3, 256] × 5	24 × 24 × 2	[3 × 3 × 1, 256] × 5
Deconvolution 1	48 × 48	3 × 3, 2 × 2-[residual structure 4]	48 × 48 × 2	3 × 3 × 1, 2 × 2 × 1-[residual structure 4]
Deconvolution 2	96 × 96	3 × 3, 2 × 2-[residual structure 3]	96 × 96 × 4	3 × 3 × 3, 2 × 2 × 2-[residual structure 3]
Deconvolution 3	192 × 192	3 × 3, 2 × 2-[residual structure 2]	192 × 192 × 4	3 × 3 × 1, 2 × 2 × 1-[residual structure 2]
Deconvolution 4	384 × 384	3 × 3, 2 × 2-[residual structure 1]	384 × 384 × 8	3 × 3 × 3, 2 × 2 × 2-[residual structure 1]
Convolutional layer	384 × 384	1 × 1, 2	384 × 384 × 8	1 × 1 × 1, 2

**Table 2:** Training set and test set information of nasopharyngeal carcinoma (NPC) segmentation model.

Data set	Number of subjects	Number of people (male/female)	Age (mean ± SD)
Training set	346	254/92	45.5 ± 11.9
Test set	75	55/20	44.9 ± 11.6

**Table 3:** Performance comparison of different NPC segmentation models.

Nasopharyngeal carcinoma segmentation model			Dice rate	HD (mm)	PAD ratio
T1W-MDF		MDF	0.77418	6.6402	20.4
T2W		MDF	0.77826	6.4974	18.258
T1C		MDF	0.76194	6.5382	20.196
T1W	T2W	MDF	0.79662	5.9568	16.83
T1W	T1C	MDF	0.78846	6.1404	17.442
T2W	T1C	MDF	0.7905	6.0486	17.136
Methods1 [20]			0.74052	6.9564	24.276
Methods2 [21]			0.73236	7.0482	25.602
Methods3 [22]			0.74562	6.885	23.154
MMMDF			0.8211	5.6712	15.81

## Data Availability

The data shall be made available on request.

## References

[1] Li Y., Dan T., Li H. (2022). NPCNet: jointly segment primary nasopharyngeal carcinoma tumors and metastatic lymph nodes in MR images. *IEEE Transactions on Medical Imaging*.

[2] Tao G., Li H., Liu L., Cai H. Detection-and-excitation neural network achieves accurate nasopharyngeal carcinoma segmentation in multi-modality MR images.

[3] Ma Z., Wu X., Zhou J. Automatic nasopharyngeal carcinoma segmentation in MR images with convolutional neural networks.

[4] Chen G., Hu H., Chen R., Xu D. Statistical classification based on SVM for Raman spectra discrimination of nasopharyngeal carcinoma cell.

[5] Zhang J., Ge Y., Chen Y., Chen X. A study on the positioning accuracy of patient positioning based on Optical Positioning System for nasopharyngeal carcinoma: Compared with conventional method.

[6] Ritthipravat P., Tatanun C., Bhongmakapat T., Tuntiyatorn L. Automatic segmentation of nasopharyngeal carcinoma from CT images.

[7] Huang K. -W., Zhao Z. -Y., Gong Q., Zha J., Chen L., Yang R. Nasopharyngeal carcinoma segmentation via HMRF-EM with maximum entropy.

[8] Zhou L. B., Zhengdong S. J., Wei D. A simple program to calculate normal tissue complication probability in external beam radiotherapy for nasopharyngeal carcinoma.

[9] Shabaz M., Garg U. (2019). Evaluation and categorization of handwriting patterns reflecting sentiments. *International Journal of Recent Technology and Engineering*.

[10] Baker O. F., Kareem S. A. ANFIS models for prognostic and survival rate analysis “nasopharyngeal carcinoma”.

[11] Gupta A., Awasthi L. K. Peer enterprises: a viable alternative to Cloud computing?.

[12] Saini G. K., Chouhan H., Kori S. (2021). Recognition of human sentiment from image using machine learning. *Annals of the Romanian Society for Cell Biology*.

[13] Kong M., Hong S. E. (2017). Tumor regression patterns by follow-up duration in patients with nasopharyngeal carcinoma treated with concurrent chemoradiotherapy. *Journal of Radiation Research*.

[14] Thakur T., Batra I., Luthra M. (2021). Gene expression-assisted cancer prediction techniques. *Journal of Healthcare Engineering*.

[15] Dai P.-s., Wang B., Chen M., Min X., Ju Y., Huang S. Computer simulation of radioactive source delivery process in nasopharyngeal carcinoma brachytherapy.

[16] Chaudhury S., Shelke N., Sau K., Prasanalakshmi B., Shabaz M. (2021). A novel approach to classifying breast cancer histopathology biopsy images using bilateral knowledge distillation and label smoothing regularization. *Computational and Mathematical Methods in Medicine*.

[17] Lu H., Lin H., Feng G. (2012). Interfractional and intrafractional errors assessed by daily cone-beam computed tomography in nasopharyngeal carcinoma treated with intensity-modulated radiation therapy: a prospective study. *Journal of Radiation Research*.

[18] Gupta A., Awasthi L. K. (2009). Security issues in cross-organizational peer-to-peer applications and some solutions. *Contemporary Computing. IC3 2009*.

[19] Li C., Niu H., Shabaz M., Kajal K. (2022). Design and implementation of intelligent monitoring system for platform security gate based on wireless communication technology using ML. *International Journal of Systems Assurance Engineering and Management*.

[20] Fung W. W. K., Wu V. W. C., Teo P. M. L. (2014). Developing an adaptive radiation therapy strategy for nasopharyngeal carcinoma. *Journal of Radiation Research*.

[21] White P., Chan K. C., Cheng K. W., Chan K. Y., Chau M. C. (2013). Volumetric intensity-modulated arc therapy vs conventional intensity-modulated radiation therapy in nasopharyngeal carcinoma: a dosimetric study. *Journal of Radiation Research*.

[22] Jiang H., Lu H., Yuan H. (2015). Dosimetric benefits of placing dose constraints on the brachial plexus in patients with nasopharyngeal carcinoma receiving intensity-modulated radiation therapy: a comparative study. *Journal of Radiation Research*.

